The article "Major trauma affecting the spine, chest wall and arm survived by a 9th/10th century CE individual from Rižinice Croatia" was published in 2024. Journal: Heliyon.

# Major trauma affecting the spine, chest wall and arm survived by a 9th/10th century CE individual from Rižinice Croatia

**DOI:** 10.1016/j.heliyon.2024.e37515

**Published:** 2024-09-05

**Authors:** Ana Curić, Fabio Cavalli, Željana Bašić, Ivana Kružić, Ivan Skejić, Krešimir Dolić, Deni Tojčić, Ivan Jerković

**Affiliations:** a Museum of Croatian Archaeological Monuments, Gunjačina 3, 21 000, Split, Croatia; b Research Unit of Paleoradiology an Allied Sciences, via della Pietà 2/1, Ospedale Maggiore, Trieste, Italy; c University Department of Forensic Sciences, University of Split, Ruđera Boškovića 33, 21000, Split, Croatia; d University Hospital Center in Split, Department of Diagnostic and Interventional Radiology, Spinčićeva 1, 21000, Split, Croatia; e University Department of Health Studies, University of Split, Ruđera Boškovića 35, 21000, Split, Croatia

**Keywords:** Antemortem trauma, *Patella cubiti*, Medieval health, Paleoradiology, Paleopathology

## Abstract

This study investigates a series of antemortem injuries in the skeletal remains of a 36-45-year-old male from the medieval site of Rižinice. It presents the injuries comprising a fractured sternum, spinal hyperflexion, multiple rib fractures, and a non-union fracture to the olecranon process of the left ulna and a *patella cubiti*, a rare anomaly, which until now has not been reported in a paleopathological context. The research aims to uncover the causes, timing, and effects of these traumata, providing insight into the challenges of life in the mid-9th to mid-10th century.

## 1 Introduction

Traumatic injuries have a highly important role in analyzing human remains from archaeological sites. By studying these injuries, we not only learn about an individual's life [[1], [2], [3]] but also obtain valuable insight into the occurrence and patterns of violence within and outside of the community. This allows us to understand the lifestyle of a specific population including tracking the occurrence and distribution of accidents and intentional violence in various environmental, cultural, or social contexts [[4], [5], [6]].

In the analysis of an individual's life, antemortem and perimortem traumata are of crucial importance. Specifically, a large proportion of peri- and antemortem traumata in a population suggests interpersonal violence and circumstances leading to accidental fractures. However, surviving major injuries may indicate to the quality of healthcare and the community's attitude towards the injured and ill [[7], [8], [9]].

Croatian medieval populations have been extensively studied for demographic, pathologic, and life-quality indicators, which also included analysis of the frequency and distribution of traumata [[10], [11], [12], [13], [14]]. However, the finding of unusual injuries and anomalies can shed additional light on the living conditions and diseases of a population.

The archaeological site of Rižinice^1^ is located northeast of Solin (ancient Salona), close to the city of Split (ancient Spalatum) (Fig. 1). At the foothills of Rižinice, flows the stream Rupotina which, in ancient times, was accompanied by a road [15]. Along this road in 1930, the remains of a Roman *villa rustica* were discovered [16]. In the oldest preserved document, dated March 4th, 852, Duke Trpimir granted this land to the Archbishop of Split as a gesture of gratitude for a loan of 11 pounds, which he needed to acquire silverware for the monastery church [16].

**Fig. 1:** The location of the archaeological site of Rižinice.

According to the document, Duke Trpimir mentioned that he had built a monastery and brought a group of brothers, or monks, into it [17]. The revelation of the monastery and the commencement of archaeological investigations at the Rižinice site were prompted by the discovery of a fragment of the altar barrier with the inscription "PRO DUCE TREPIME(ro)." The initial explorations were conducted in 1895 by the "Bihać" society. A small single-nave church with a semicircular apse and a vestibule, measuring a total of 16 x 7.4 m,^2^ oriented north to south, were uncovered. The presbytery area was spacious, suggesting that the church had been primarily intended for the clergy [15]. On the west side of the church monastery, rooms were positioned, and around the church was a cemetery with a rich history of burials, spanning from 2nd to 3rd century AD to the era of the Venetian Republic [16]. After the investigations at the end of the 19th and the beginning of the 20th centuries, the site was explored by the Institute for the Protection of Cultural Monuments, and later, the Museum of Croatian Archaeological Monuments (MHAS) in Split [18].

In 2021, the MHAS conducted archaeological research, exploring 54 graves from the mid-9th to the mid-10th century (Fig. 2), which were dated by analogies of archaeological artifacts found within them, for example, single-bead earrings [18]. The graves, made of stone with lining, headstone, footstone, and tomb cover, were grouped based on their orientation. Many graves were disturbed by past excavations, with skeletal remains that were not in their original positions. As males, females, and non-adults were buried in the cemetery, it most likely belonged to the local population. Grave 3, located at the eastern edge, was undisturbed. It contained the remains of four individuals, including a non-adult with the least preserved skeletal remains, alongside well-preserved remains of a female and two male individuals [19] (Fig. 3).

**Fig. 2:** Aerial view of the explored site. North of the graves are the remains of a Benedictine monastery with a single-nave church, while to the east are the remains of a Roman villa rustica.

**Fig. 3:** Photograph and sketch. Skeletal remains of interest are highlighted. Yellow represents plaster and orange ceramics.

In this study, we will provide a detailed description of the traumata and pathology identified in a male individual from grave 3 who was the first to be interred in the grave. We will also explore the possible mechanisms behind their occurrence, examine the circumstances that could have led to the injuries using anthropological and radiographic analysis, and investigate life after injury and the support of society.

## 2 Materials and methods

### 2.1 Anthropological analysis

In the laboratory, the osteological material retrieved from the site was washed under a gentle stream of water and left to air dry. After positioning remains into their anatomical position and assessing the degree of preservation [20,21], the biological profile of each person was estimated. Following the anthropological analysis, the bones were documented and photographed. Anthropological assessment of sex was made based on the morphology of the pelvis (overall morphology, greater sciatic notch) and skull (overall skull and mandible morphology, glabella, nuchal crest, mastoid process) [21,22]. Age was estimated by changes in the pubic symphysis [23,24], and auricular surface [25], along with examination of degenerative changes of the joints [22] and dental wear [26]. The skeleton was visually inspected and examined for pathological and traumatic changes [27]. We also examined the remains and discovered the most common skeletal pathology, such as cribra orbitalia [28], otitis media [29,30], degenerative joint disease [31,32] and periosteal new bone formation [33,34]. Stature was estimated using the maximum length of the femur and the formula developed by Ruff et al. [35].

### 2.2 Radiographic analysis

Following the anthropological analysis, bones with pathological lesions underwent multi-slice computed tomography (MSCT) scanning at the Department of Diagnostic and Interventional Radiology, University Hospital Center in Split, Croatia. The scanning procedure employed the MSCT device model SOMATOM go. TOP (manufactured by Siemens Healthineers, Germany). The scan was conducted with the following specifications: 100 kV and 57 mA, with a slice thickness of 0.6 mm. Firstly, the bones were carefully placed on radiolucent support, specifically a piece of expanded polystyrene. Following this, separate scans of the sternum, ribs, two thoracic vertebrae, and the left ulna and radius were taken. None of the bones were overlapping or articulated with each other. Images were examined by an experienced paleoradiologist (FC) and skeletal structures of interest were measured. Image processing and analysis were performed using RadiAnt DICOM Viewer (Medixant, Poland) and the SuitExtensa PACS Enterprise system (ESAOTE s.p.a., Genova), with 3D reconstructions generated through Autodesk 3D Studio Max (Autodesk Inc., St Rafael, CA, USA).

## 3 Results

The oldest individual in Grave 3 was a well-preserved male skeleton aged 36–45 at the time of death, with an estimated stature of 171.5 ± 3.2 cm. The postcranial skeleton was complete, the cranial skeleton consisted of a preserved calvarium and mandible, but the splanchnocranium was absent.

The skeleton displayed bilateral porosity of the orbital roof and bilateral perforations on the temporal bones with evidence for remodelling (both in the final stage of healing). Osteophytes, porosity, and hypertrophy of the facet joints were visible on all cervical and lumbar vertebrae. Osteophytes were also visible on the proximal femora and elbow joints, as well as the distal tibiae. Additionally, periosteal new bone formation, with newly formed lamellar bone, was visible on the distal femora epiphyses, distal tibiae epiphyses, and medial tibial shaft.

The skeleton exhibited antemortem traumata (indicated by bone healing), including injuries to the sternum, ribs, compression injuries to the spine, and an injury to the left ulna. All the fractures had been healed at the time of death, without traces suggesting peri-mortem injuries.

Anthropological analysis revealed a bipartite sternum. The superior segment consisted of the manubrium fused to the proximal half of the *corpus sterni*, with a transverse fracture between the second and third sternebrae (Fig. 4). The inferior segment comprised the distal *corpus sterni* and the fused xiphoid process.

**Fig. 4:** Sternum, schematic articulation of fragments (3D reconstruction from CT): a.) anterior b.) lateral c.) posterior oblique.

Malunion occurred with significant overlap of the inferior segment onto the superior segment, resulting in a pseudoarthrosis at the point of overlap rather than the original fracture site. Consequently, the majority of the superior *corpus sterni* was positioned posterior to the inferior segment. Subsequent CT imaging confirmed these findings and demonstrated posterior displacement of the caudal two-thirds of the sternum due to disruption of the articulation between the second and third sternebrae (Fig. 4, Fig. 5). This displacement led to the formation of a new joint, ultimately causing shortening and deformity of the sternum. The length of the sternum's cranial part was 10.7 cm and of caudal 8.9 cm. When parts of the sternum overlapped and were positioned as such over the lifetime (Fig. 4), total sternal length was 17.1 cm.

**Fig. 5:** CT MIP (maximum intensity projection) reconstruction: visible sternebral ossifications with drawing and photograph of the broken sternum.

In addition to an antemortem fracture of the sternum, bone calluses were found on the left 4th, 5th, and 8th ribs, as well as the right 3rd, 5th, and 9th ribs with no evidence of infection. All of the calluses were located at the superior parts of the ribs’ angles (Fig. 6).

**Fig. 6:** Photography and CT scan, MIP reconstruction (maximum intensity projection). Left 4th and 5th rib fractures, posterior aspect (asterisk).

Also, antemortem changes were found to the 5th and 8th thoracic vertebrae bodies, characterized by structural destruction (collapse). In contrast, the 3rd and 4th thoracic vertebrae showed less severe compression (Fig. 7).

**Fig. 7:** CT orthogonal sections of T5 (a.) & T8 (b.) 3D reconstruction; 1. coronal, 2) axial, 3) sagittal.

Besides the injuries previously mentioned, the proximal part of the left ulna also exhibited trauma. There was a separation of the olecranon process, occurring proximal to the height of the coronoid, characterized by an oblique fracture line sloping on the posterior/inferior side. A pseudarthrosis was formed at the point of contact between the displaced olecranon and the rest of the bone (Fig. 8). Finally, there was a bone fragment that had been separated from the olecranon process of the left ulna, displaying a resemblance to the shape of a patella (dry bone dimensions: 2.8 × 1.5 cm) (Fig. 8). The examination unveiled an articular surface and olecranon process without any unusual traits and dimensions. Upon comparison with the opposite side of the body, both elbow joint surfaces were found to be similar in size.

**Fig. 8:** Left ulna, schema (3D reconstruction from CT scan). 1) *Patella cubiti*; 2) Olecranon with fracture and pseudoarthrosis with 3) distal portion of ulnar epiphysis.

## 4 Discussion

This study analyzed two very rare skeletal conditions in the archaeological context: uncommon sternal injury with pseudoarthrosis and *patella cubiti.* The rarity of these findings are important for both clinicians and paleopathologists. The clinicians could benefit from the aspect of posttraumatic recovery without intervention as well as studying a case that is not common in today's practice. The finding of *patella cubiti* adds to the existing knowledge about this anomaly. In regard to paleopathologists and anthropologists, this study can give insight into traumata survival, the ways of their interpretation, and about life after the “event”.

The fractures appear to have occurred at a *locus minoris resistentiae*, specifically within sternebrae that had not yet fused. This could indicate that the trauma occurred during adolescence or early adulthood, as sternebrae typically fuse with age. Despite the sternum shortening due to the trauma, where the lower portion shifted anteriorly relative to the upper portion, the overall length of the sternum, excluding any overlapping bone segments, exceeded the typical length found in adult male Croatian sterna, where the average manubrium was ca. 6 cm and the sternal body 10 cm in length [36]. In contrast, the total length of the sternum in this study was 17.1 cm with pseudoarthrosis and 19.6 cm in total (non-anatomical) length. This supports our assumption of the trauma during growth as fractures in such cases can exhibit longitudinal bone growth causing the adult bone to be longer than it could have been without trauma occurring [37].

Sternal fractures are primarily caused by direct injury [38], such as a blow to the chest or accidents involving compression, falls from heights, or spinal hyperflexion [39,40]. When a blow impacts the upper part of the sternum, the manubrium (top section of the sternum) is pushed backward. The backward movement is due the upward and outward motions of the lower part of the sternum, which is influenced by the movement of the lower ribs, diaphragm, and abdominal organs during breathing. The clavicle and first rib exert downward pressure on the upper part of the sternum. Conversely, if the blow strikes the lower sternum, the inferior section is displayed posteriorly, while the upper section remains supported by the clavicles and first ribs. Such impacts are often accompanied by rib fractures [39]. All bone calluses present on the ribs were located on the posterior side which is the most common position of rib fractures caused by the indirect force [40]. This could indicate that the direct force was inflicted on the chest, broke the sternum, and indirectly fractured the ribs. A direct blow to the sternum that resulted in hyperflexion could have also caused damage and destruction of the vertebral bodies [41]. In this case, the 5th and 8th thoracic vertebrae while the 3rd and 4th thoracic vertebrae experienced less severe compression forces.

Rib fractures are the most commonly associated injury to sternal injuries, with spinal fractures being the second most frequent [42]. Secondary injuries, such as broken ribs and compression injuries of the spine, indicate that the injury likely did not occur when the person was in early childhood. Sternum trauma in young children usually does not cause damage to the ribs and spine since children's bones are very flexible, therefore protecting them from fractures and injuries [43]. The first fusion of the sternum occurs among 3rd and 4th sternebrae at ages between 4 and 15, while 2nd sternebrae fuse by the age of 11–20. The last sternebrae to fuse is the first one, which occurs around 15–25 years. An exception to this is the xiphoid process which fuses later in life [22]. This is particularly notable as vertebrae and rib fractures during this period tend to exhibit a distribution pattern like that observed in adults. These cases typically result in long-term consequences and lack the potential to remodel the deformed vertebral body [44]. When the spine bends, the clavicles, ribs, and sternum move down and position behind the lower part of the sternum. This can cause the upper and middle parts of the thoracic spine to curve forward [45]. Such displacement of the lower fragment can cause visible and palpable ridge-like deformities near the fracture. During these injuries, the posture is often described as having the head and body bent forward. Recovery with bone callus formation typically takes four to eight weeks, but permanent deformation may occur to some extent [46].

Regarding the left elbow, antemortem trauma on the proximal ulna is a common arm injury [47], mainly caused by direct trauma, for example, falls with force applied on the dorsal side of the elbow [48] or falls on an outstretched hand when the triceps contraction causes the injury. When forces generated by the arm muscles (triceps, biceps, and brachialis) are too strong or unbalanced, they can pull on the bones in a way that makes the misalignment of the joints even more severe [47]. The remaining part of the ulna was intact, with no changes visible on diaphysis, distal articular surface, nor in bone length.

The left distal humerus and proximal radius showed no signs of injury, deformity, or muscle overuse. The absence of secondary trauma and pathological changes on the bones of the left arm could indicate that the injury occurred while the person was still growing. Specific data obtained from modern cases of olecranon fractures, for the injuries sustained before the age of 16, indicate that they do not lead to deformations and exceptional pathological changes in later life [49].

Besides the trauma found on the ulna, it is important to mention a bone fragment separated from the left ulna, exhibiting a sharp edge, which created the appearance of a discontinuous joint line [50]. The smooth and regular bone edges with a cortical outline on both sides indicate that the elbow was neither partially nor fully dislocated [51]. Since the joint surfaces of the right and left elbow joints are similar, an old injury cannot account for this type of olecranon displacement [50]. Hence, we can infer that this is a case of *patella cubiti*, a rare abnormality impacting the elbow, where either the entire olecranon or a portion remains detached from the proximal ulna. The cause of this condition remains uncertain due to its rarity, with various hypotheses put forward, including congenital [52], developmental [53], and traumatic origins [54]. This anomaly typically accompanies pain and stiffness, along with a reduction in stretching ability and disability, although some patients do not exhibit any symptoms [51].

An analysis of 18 modern cases of *patella cubiti*, reveals its occurrence in both males and females, affecting individuals across subadult and adult age groups. In most instances, the anomaly manifests as pain and limited elbow mobility, and with no association to prior elbow injuries. The current treatment approach for *patella cubiti* involves surgical intervention [51]. Notably, this anomaly has not been documented in paleopathological records to date, and the prevalence in one studied modern population was 0.79 % (13 in 1646 people) [55]. In conjunction with the large fracture of the olecranon process of the left ulna, this anomaly most likely contributed to pain and reduced mobility of the left elbow.

Based on the anthropological and radiological analysis of the severe injuries sustained by the male individual from Grave 3, it is evident that he experienced significant trauma during his adolescent years (according to Ref. [56] adolescent period ranges from 13 to 20 years) or early adulthood. These traumata may have had a lasting impact on his life, such as visible sternum protrusion and the forward-leaning gait caused by hyperflexion of the spine [46].

Considering the impact of described conditions on the individual's life, the injuries could have resulted in restricted mobility, chronic pain, and could have impacted some daily or routine activities of the individual. Also, this individual likely obtained these injuries while he was still developing which would have required physical and psychological care and support, assistance with mobility, and likely an adequate diet that facilitates healing. The healed injuries could have demonstrated that the community had a certain level of knowledge and resources to provide long-term care. The burial in a communal grave and the attention to the individual's injuries could indicate a society that valued and took responsibility for its members, and also to an individual who likely adapted to his limitations and found a way to contribute to the society.

## 5 Conclusion

This study pointed out the necessity of interdisciplinary collaboration of different experts, for example, archaeologists, anthropologists, and clinicians (radiologists) in studying paleopathological conditions and interpreting past events, especially in the context of individual history and the interpretation of the social context. Although we could not give conclusions about the mechanisms of traumata and exact time sequence, we could estimate the most probable sequence of events and trauma mechanisms. By the analysis of the overall health of the individual, we could argue about the level of the healthcare and general relation of the society towards that person, and *vice versa*.

## Funding

None.

## Data availability statement

MSCT images of the specimen are available upon reasonable request.

## Ethical statement

The issues regarding informed consent and ethical approvals are not applicable in the present study as it analyzed a skeleton from an archaeological context.

## CRediT authorship contribution statement

**Ana Curić:** Writing – review & editing, Writing – original draft, Visualization, Resources, Methodology, Investigation, Formal analysis, Conceptualization. **Fabio Cavalli:** Writing – review & editing, Writing – original draft, Methodology, Investigation, Formal analysis, Conceptualization. **Željana Bašić:** Writing – review & editing, Writing – original draft, Supervision, Resources, Methodology, Conceptualization. **Ivana Kružić:** Writing – review & editing, Resources, Methodology, Investigation, Conceptualization. **Ivan Skejić:** Writing – review & editing, Resources, Methodology, Investigation, Conceptualization. **Krešimir Dolić:** Writing – review & editing, Resources, Methodology, Investigation, Conceptualization. **Deni Tojčić:** Writing – review & editing, Resources, Methodology, Investigation, Conceptualization. **Ivan Jerković:** Writing – review & editing, Writing – original draft, Supervision, Resources, Methodology, Investigation, Conceptualization.

## Declaration of competing interest

The authors declare that they have no known competing financial interests or personal relationships that could have appeared to influence the work reported in this paper.

## Footnotes

1 Coordinates of the archaeological site: 43.55520250205875, 16.498875026240604 l.

2 New research suggests that the dimensions of the church were, in fact, 12.97 × 7.4 m, but the studies have not yet been published (DT).
